RETRACTED

# Long non-coding RNA DCST1-AS1/hsa-miR-582-5p/HMGB1 axis regulates colorectal cancer progression

**DOI:** 10.1080/21655979.2021.1976894

**Published:** 2021-12-30

**Authors:** Long huang, Gang Dai

**Affiliations:** a Department of General Surgery, Beibei Traditional Chinese Medical Hospital, Chongqing, China; b Department of General Surgery, Fengdu People’s Hospital, Fengdu County, Chongqing, China

**Keywords:** DCST1-AS1, CRC, hsa-miR-582-5p, HMGB1

## Abstract

Long non-coding RNAs (lncRNAs) are related to the initiation and progression of tumor and regulate various cellular processes including growth, invasion, migration, and apoptosis. Understanding the roles and mechanisms of lncRNAs in regulating cancer progression is crucial for formulating novel therapeutic strategies. Although lncRNA DCST1-antisense RNA 1(AS1) has been implicated in several cancers, its role in the progression of colorectal cancer (CRC) remains to be explored. This study focuses on elucidating the function of lncRNA DCST1-AS1 in CRC development and its underlying mechanism. We found that the expression of lncRNA DCST1-AS1 was up-regulated in CRC tissues and cell lines, and CRC patients with high lncRNA DCST1-AS1 expression were associated with a poor prognosis. Loss-of-function and gain-of-function experiment in CRC cell lines confirmed that lncRNA DCST1-AS1 promoted the malignant phenotype of CRC cells, including cell proliferation, colony formation, migration, and invasion. In addition, we identified the binding sites between lncRNA DCST1-AS1 and hsa-miR-582-5p, and between hsa-miR-582-5p and High Mobility Group Box 1 (HMGB1) through DIANA Tools and TargetScan database, which was further confirmed by dual-luciferase reporter assay. Functional assay further confirmed the crucial role of lncRNA DCST1-AS1/hsa-miR-582-5p/HMGB1 axis in modulating the malignant phenotype of CRC cells. Collectively, our data suggest that lncRNA DCST1-AS1 regulates the aggressiveness of CRC cells through hsa-miR-582-5p/HMGB1 axis. Our study provides novel insight into the mechanism of lncRNA DCST1-AS1 in CRC cells for targeted therapy.

## Introduction

Colorectal cancer (CRC) is third most common cancer worldwide, which accounts for approximately 10% of annual cancer cases globally [1,2]. Accumulating evidence shows that CRC is a highly heterogeneous tumor with different molecular and clinical characteristics, indicating the necessity of personalized treatment [3]. Chemotherapy and surgery are the main therapeutic strategies for CRC [4]. For patients with advanced CRC, surgery combined with chemotherapy and radiotherapy is a more effective strategy for CRC patients [5,6]. Recent improvements in combinatory chemotherapy and the development of targeted therapies have improved the overall survival (OS) rate among advanced CRC cases. Nonetheless, drug resistance poses a major challenge for effectively eradicating cancer cells in CRC patients [7–9]. As a result, understanding the mechanisms underlying poor CRC prognosis at molecular level is important, which holds the promise for novel therapy development.

RETRACTED

Non-coding RNAs (ncRNAs), which include microRNAs (miRNAs) and long ncRNAs (lncRNAs), regulate gene expression and are implicated in cancer progression [10]. LncRNAs are a class of ncRNAs with over 200 nucleotides in length and they have little protein-coding capacity [11–13]. Evidence mounts that aberrant lncRNA expression facilitates malignant tumor progression, and targeting lncRNAs draws increasing attention as a targeted cancer therapy [10,14,15]. However, the roles and functions of most lncRNAs are still unclear. LncRNA DCST1 antisense RNA 1 (DCST1-AS1) is identified as an oncogenic lncRNA in malignant tumors like hepatocellular carcinoma (HCC) and breast cancer (BC) [16–18]. Its potential role and regulatory mechanisms in CRC remain to be clarified. miRNAs, a short ncRNA molecule containing about 22 nucleotides, regulate gene expression by targeting mRNA [19]. miRNAs are involved in many cellular processes including cellular growth and metastasis [20–22]. Among them, hsa-miR-582-5p is recognized as the tumor suppressor in prostate cancer (PCa) and non-small cell lung cancer (NSCLC) [23,24]. In many scenarios, lncRNAs can competitively bind to miRNAs and inhibit their activity, thereby regulating the expression of the downstream target genes [17].

High-mobility group box-1 (HMGB1), one of the highly conserved nuclear proteins [25], is involved in the regulation of inflammatory response [26] and sepsis-induced acute lung injury [27]. HMGB1 has also been implicated in progression of different types of cancers, which serves as a novel biomarker for tumor diagnosis and treatment [28]. For example, HMGB1 enhances lymph node metastasis (LNM) in esophageal squamous cell carcinoma (ESCC), with HMGB1 upregulation being associated with a poor prognosis [29]. In hepatocellular carcinoma, high HMGB1 expression is also linked to a poor prognosis [30]. In CRC patients, HMGB1 expression is also proposed as a prognostic marker related to CRC patient survival [31,32]. A recent study revealed that HMGB1 is also implicated in papillary thyroid carcinoma progression [33]. However, the mechanisms regulating HMGB1 expression in CRC remains to be elucidated.

The present work aims to explore the potential role of lncRNA DCST1-AS1 in modulating CRC cell phenotype and the underlying mechanisms. We compared the expression of lncRNA DCST1-AS1 between CRC tissues and normal tissues adjacent to cancer, as well as the expression between CRC cells and non-carcinoma colonic epithelial cells. A significantly higher expression of lncRNA DCST1-AS1 was observed in CRC tissues and cell lines, which was associated with a poorer overall survival of CRC patients. The above results suggested the oncogenic effect of lncRNA DCST1-AS1 in CRC. Loss-of-function and gain-of-function experiments in CRC cell lines confirmed the oncogenic role of lncRNA DCST1-AS1 to promote the malignant phenotype of CRC cells. We further identified hsa-miR-582-5p as a binding partner of lncRNA DCST1-AS1. By negatively regulating the activity of hsa-miR-582-5p, lncRNA DCST1-AS1 enhances the expression of HMGB1 to promote the aggressiveness of CRC cells. Collectively, our data demonstrated the role of lncRNA DCST1-AS1/hsa-miR-582-5p/HMGB1 axis in modulating the malignant phenotype of CRC cells. Our study provides novel insight into the mechanism of lncRNA DCST1-AS1 in CRC cells for targeted therapy.

RETRACTED

## Materials and methods

### Tissue samples

A total of 60 pairs of CRC tissues and the matched adjacent normal tissues were collected in Fengdu People’s Hospital of Chongqing (Chongqing, China) from January 2017 to December 2019. CRC patients enrolled in the study did not experience radiotherapy and chemotherapy before surgery. This study was approved by the Medical Ethics Committee of Fengdu People’s Hospital of Chongqing (Approval number: CQSHIRB-K-20200405), and the written informed consent form was signed by all patients. All the samples were collected by surgery and stored in the refrigerator at −80°C until further analysis.

### Cell culture, transfection, and lentivirus infection

CRC cell lines SW620, HCT116, LoVo, colo205, HT-29 and SW480, and normal human colonic epithelial cell NCM460 cells were obtained from Cell Bank of Chinese Academy of Sciences (Shanghai, China). Cells were routinely cultured in DMEM medium containing 10% fetal bovine serum (Thermo Fisher Scientific/Gibco, Gaithersburg, MD, USA) and supplemented with 100 U/ml penicillin and 100 mg/ml streptomycin (Invitrogen, Carlsbad, CA, US) in a humidified incubator under the condition of 37°C and 5% CO_2_.

The recombinant lentivirus carrying short hairpin RNA (shRNA) targeting lncRNA DCST1-AS1 and its negative control were prepared by Shanghai Genechem Co., Ltd (Shanghai, China). HT-29 CRC cells were infected with the recombinant lentivirus at a MOI (multiplicity of infection) of 5 in the presence of 10 µg/ml polybrene (Sigma, tr-1003-g). Infected cells were selected with 1.0 μg/mL puromycin for two weeks to eliminate the uninfected cells before further experiment. qPCR was performed to confirm the efficient knockdown of lncRNA DCST1-AS1.

hsa-miR-582-5p inhibitor, hsa-miR-582-5p mimic, the corresponding controls, pcDNA3.1-DCST1-AS1 construct, pcDNA3.1-HMGB1 construct, negative control (NC) plasmid and siRNAs were synthesized and purchased from RiboBio Co, Ltd. (Guangzhou, China). Transfection was performed using Lipofectamine 3000 (Invitrogen, L3000001) according to the manufacturer’s instructions. 50 nM of each molecule or 5 µg of plasmid was used for transfection, and functional experiments were performed 48 hours post-transfection.

RETRACTED

### RT-qPCR

RT-qRCR was conducted according to the method described in previous study [34]. TRIzol reagent (Invitrogen) was used for extracting total RNA, and the concentration and purity of the purified RNA was measured by NanoDrop. 5 μg total RNA was used for reverse transcription by SuperScript First Strand cDNA System (Invitrogen). Then, SYBR premix EX TAQ II (Takara, Dalian, China) was used to perform real-time qRCR on the 7500 Real-Time PCR System (Applied Biosystems/Life Technologies, Carlsbad, CA, USA). The results were analyzed using 2^–∆∆Ct^ method and glyceraldehyde-3-phosphate dehydrogenase (GAPDH) was used as the endogenous control. Primer sequences were synthesized by Shanghai Sangon Biotechnology Co., Ltd. (Shanghai, China) as follows: lncRNA DCST1-AS1 (5'- TTCGTCTGGTCCCAATGTGTGG-3', forward; 5'-AAGCAGGACGAGTAAACCA ACC-3', reverse); GAPDH (5'-CATGAGAAGTATGACAACAGCCT-3', forward; 5'-AGTCCTTCCACGATACCAAAGT-3', reverse); Hsa-miR-582-5p (5'-GCGGTTACAGTTGTTCAACC-3', forward; 5'-CTCAACTGGTGTCGTGGA-3', reverse);HMGB1 (5'-TATGGCAAAAGCGGACAAGG-3', forward; 5'- CTTCGCAACATCACCAATGGA −3', reverse).

### CCK8 cell proliferation assay

Changes in cell proliferation were detected by CCK8 assay. CRC cells were seeded into a 96-well plate at a density of 1 × 10^4^ cells/well, and incubated in a 37°C cell culture incubator containing 5% CO2 for desired period. 10 μL CCK-8 reagent was added to each well at indicated time point and incubated in the incubator for 1 hour. The GX71 microplate reader (Olympus Japan) was used to detect the absorbance value (OD value) in each well at 450 nm [35].

### Colony formation assay

Colony formation assay was used to evaluate the long-term proliferation potential of HT-29 and HCT116 cells. Cells were infected with recombinant lentivirus carrying shRNA targeting lncRNA DCST1-AS1 or co-transfected with miR-582-5p-inhibitor (inh) or pcDNA3.1-HMGB1 or their corresponding controls. Forty-eight hours post-transfection, cells were seeded into a 6-well plate at the density of 200 cells/well. The culture medium was changed every two days. After 14 days’ culture, cells were fixed with 4% paraformaldehyde and stained using Giemsa Stain Kit (Abcam, ab150670) according the manufacturer’s instructions. Finally, the number of colonies formed in each condition was counted using Leica AM6000 microscope [36].

RETRACTED

### Cell invasion and migration assay

For the invasion assay, Matrigel (354,230, BD, USA) was diluted in an appropriate proportion and coated on the bottom of transwell chamber (CLS3398, Sigma, Germany). For the migration assay, Matrigel was not used. Cells were trypsinized and then resuspended in serum-free medium. After cell counting, 1 × 10^4^ cells were seeded into the upper chamber in medium with 3% FBS, and 500 μL medium with 10% FBS was added into the lower chamber. The cells were cultured in incubator for 48 hours, followed by fixation with 4% paraformaldehyde for 10 mins at room temperature and staining with 0.5% crystal violet solution (c0755, Sigma, Germany) in 25% methanol for 20 minutes. The invading and migrating cells were imaged and counted using Leica AM6000 microscope [37].

### Xenograft tumorigenesis assay

HT-29 cells (5 × 10^6^) that stably expressing lncRNA DCST1-AS1 shRNA (sh-lncRNA DCST1-AS1#1) or the control shRNA(sh-NC) were subcutaneously inoculated into the 6 weeks old BALB/c nude mice. The tumor volume and weight were measured continuously for 5 weeks. The mice were sacrificed on days 40 and the tumors in the mice were extracted. The formula V = (width^2^ x length/2) was used to calculate the tumor size. All experimental procedures of animal study were approved by the Laboratory Animal Ethics Committee at Chongqing Fengdu People’s Hospital.

### Immunohistochemistry (IHC)

Immunohistostaining of Ki-67, N-Cadherin and E-Cadherin was performed on 4-mm sections of formalin-fixed paraffin-embedded (FFPE) tumor tissue. First, deparaffinization and hydration were performed by sequentially incubating the section in xylene for 5 min, in 100% ethanol for 10 min, in 95% ethanol for 10 min, and in dH_2_O for 5 min. The section was submersed in 1X citrate unmasking solution (SignalStain® Citrate Unmasking Solution (10X), Cell Signaling Technologies, #14,746) for heating in a microwave at a sub-boiling temperature (95°–98°C) for 10 mins. After cooling, the sections were washed in dH_2_O and incubated in 3% hydrogen peroxide for 10 min. Then, the section was blocked with 5% Normal Goat Serum for 1 hour at room temperature. The primary antibodies Ki-67 (D3B5, #9129), E-Cadherin (24E10, #3195) and N-Cadherin (D4R1H, #13,116) (Cell Signaling Technologies) were diluted 1:500 in TBST buffer, and the section was incubated with the primary antibody overnight at 4°C. The section was washed three times using TBST buffer. The section was soaked with 1–3 drops SignalStain® Boost Detection Reagent (HRP, Rabbit, Cell Signaling Technologies, #8114) and incubated in a humidified chamber for 30 min at room temperature. 200 µL SignalStain® substrate (Cell Signaling Technologies, #8059) was added to each section for 5 min incubation. The section was washed in dH_2_O two times for 5 min each and then dehydrated. Section was mounted with coverslips in the mounting medium (Cell Signaling Technologies, #14,177) before imaging [38].

RETRACTED

### Dual-luciferase reporter assay

To demonstrate the functional interaction between lncRNA DCST1-AS1 and miR-582-5p, the sequence containing the wild type binding site and the sequence with mutated binding site of lncRNA DCST1-AS1 were cloned into the PmirGLO vector expressing firefly luciferase, respectively (Promega, E1330). The reporter plasmid and Renilla luciferase (hRlucneo) control plasmid were co-transfected into HT-29 and HCT116 cells with either miR-582-5p mimic or miR-NC in a 12-well plate (1 × 10^5^ cells/well) using Lipofectamine 3000 reagent according to the manufacturer’s instructions (Invitrogen, L3000001). Similarly, the reporter vector containing the wild type binding site of HMGB1 and the sequence with mutated binding site were also constructed and co-transfected with Renilla luciferase (hRlucneo) control plasmid in the presence of miR-582-5p mimic or miR-NC. 48 h post transfection, the relative luciferase activities were measured using Dual-Luciferase Reporter Assay Kit (Promega, E1910) on a luminescence microplate reader (Infinite 200 PRO; Tecan). The relative firefly luciferase activity in the reporter plasmid was normalized to that of Renilla luciferase (hRlucneo) control plasmid [39].

### RNA pull-down assay

Cells lysates were collected by IP lysis buffer (Beyotime, P0013) and were incubated with Biotin-labeled lncRNA DCST1-AS1 probe or control probe for 6 hours at 4°C. 10% of the total lysates were saved as the input. The mixture was further incubated with M-280 streptavidin magnetic beads (Sigma–Aldrich, 11205D) at 4°C shaking overnight. A magnetic bar was used to pull down the magnetic beads and associated nucleic acids, then the samples were washed 4 times with high salt wash buffer. Both the input and the elutes from the pull-down were purified with Trizol reagent (Invitrogen, 15,596,026) according to the manufacturer’s protocol. The reverse transcription was carried out using Superscript III transcriptase (Invitrogen, 18,080,093) and quantitative RT-qPCR analysis was performed using Maxima SYBR Green/ROX qPCR Master Mix (Thermo Fisher Scientific, K0221) on a LightCycler® 96 real-time PCR system (Roche) [40].

RETRACTED

### Western blotting (WB)

Western blot was used to detect protein expression level according to a previous study [37]. 70% confluent cells in 6-well plate was lysed with RIPA lysis buffer, and then centrifuged at 15,000 × g in a 4°C to remove cell debris. The protein concentration was measured using a BCA kit (Thermo, Shanghai, China). 10 ug protein was used for SDS-PAGE analysis. Separated protein in SDS-PAGE gel was transferred onto the PVDF membrane (BioRed, USA). After blocking with 5% skimmed milk for 1 hour, the membrane was then incubated with primary antibodies: anti-HMGB1 (CST, #6893, 1:1000 dilution in TBST) and anti-GAPDH (CST, #5174, 1:1000 dilution in TBST) antibodies. The primary antibodies were incubated overnight at 4°C, and the protein-loaded PVDF membrane was washed 3 times with TBST for 5 minutes each. After wash, the membrane was further incubated with HRP-labeled secondary antibody (ProteinTech, SA00001-2, 1:5000 dilution in TBST) for 1 hour. Then, the membrane was washed 4 times with TBST and protein band development was performed using Clarity ECL Western Blotting Substrates (1,705,060, Bio-Rad). ImageJ software was used to perform grayscale analysis using GAPDH as an internal reference protein.

### Bioinformatics prediction

To identify the potential-binding partners of lncRNA DCST1-AS1, we first retrieved the sequence of lncRNA DCST1-AS1 (known as RP11-307C12.11) in NCBI database (https://www.ncbi.nlm.nih.gov/gene/100505666). The sequence of lncRNA DCST1-AS1 was subject to miRNA target prediction using LncBase version 2 Prediction Module of DIANA Tools (http://carolina.imis.athena-innovation.gr/diana_tools/web/). The following search criteria were used: ‘search by location’ – enter ‘chr1:155,045,191–155,046,118’ (obtained from ensemble database http://asia.ensembl.org/ – click ‘human’ – enter ‘DCST1-AS1’) and selected ‘based on transcripts’. The threshold was set to ‘0.7’. To identify the target of hsa-miR-582-5p, TargetScan database (http://www.targetscan.org/vert_72/) was used to predict the mRNA targets containing potential-binding sites for hsa-miR-582-5p.

### Statistical analysis

Statistical analyses were conducted by SPSS13.0 (SPSS Inc., Chicago, IL, USA), while graphs were plotted using GraphPad Prism 6.0 (https://www.graphpad.com/). The data were presented as the mean ± standard deviation (SD). Student’s t test was used to compare the difference between treatment group and control group. Comparisons of continuous variables among multiple groups were analyzed using one-way analysis of variance (ANOVA). Comparisons of data at multiple time points were examined using repeated-measurement ANOVA. Kaplan–Meier and log-rank test were applied in comparing the cumulative survival rates. Pearson correlation analysis was used to assess the correlation between the expression levels of two molecules in CRC. All statistical analysis was performed using SPSS version 13.0 software. *P* < 0.05 was considered statistically significant.

RETRACTED

## Results

The purpose of this study is to elucidate the role and underlying mechanism of lncRNA DCST1-AS1 in regulating the phenotype of CRC cells. We first compared the expression of lncRNA DCST1-AS1 between CRC tumor tissues and normal tissues adjacent to cancer, as well as its expression between CRC cells and non-carcinoma colonic epithelial cells. LncRNA DCST1-AS1 was significantly upregulated in CRC tissues and cell lines, which was associated with a poorer overall survival of CRC patients. Loss-of-function and gain-of-function experiment in CRC cell lines demonstrated the oncogenic role of lncRNA DCST1-AS1 in promoting the malignant phenotype of CRC cells. We further identified hsa-miR-582-5p as a binding partner of lncRNA DCST1-AS1. By negatively regulating the expression of hsa-miR-582-5p, lncRNA DCST1-AS1 enhances the expression of HMGB1 to promote the aggressiveness of CRC cells. Collectively, our data suggest that lncRNA DCST1-AS1/hsa-miR-582-5p/HMGB1 axis plays an important role in modulating the malignant phenotype of CRC cells.

### LncRNA DCST1-AS1 is significantly up-regulated in colorectal cancer tissues and cell lines

In order to explore the role of lncRNA DCST1-AS1 in the progression of CRC, qRT-PCR was used to detect the expression levels of lncRNA DCST1-AS1 in CRC tumor tissues and the paired adjacent normal tissues from 60 patients. We found that the expression level of lncRNA DCST1-AS1 was significantly higher in CRC tissues (Figure 1a). Consistently, lncRNA DCST1-AS1 displayed a higher expression in CRC cell lines SW620, HCT116, LoVo, colo205, HT-29, SW480 when compared to that in normal human colonic epithelial cells NCM460 (Figure 1b). Next, we took the median expression value of lncRNA DCST1-AS1 in CRC tissue in Figure 1a as the cutoff to divide 60 CRC patients into high (n = 30) or low (n = 30) expression group. Kaplan–Meier survival curve was employed to evaluate overall survival rate of two groups of patients. Our analysis showed that the prognosis of patients with high level of lncRNA DCST1-AS1 was significantly poorer (Figure 1c). Collectively, the above findings suggest the possible role of lncRNA DCST1-AS1 as an oncogenic factor that promotes the progression of CRC.

**Figure 1.** **Elevated expression level of lncRNA DCST1-AS1 within CRC cells and tissues.** (a) The lncRNA DCST1-AS1 levels within 60 pairs of CRC samples and non-carcinoma samples were measured through RT-qPCR. (b) RT-qPCR was conducted to detect lncRNA DCST1-AS1 levels within CRC cells (HCT116, SW620, colo205, LoVo, SW480, HT-29) and non-carcinoma human colonic epithelial cells (NCM460). The above results were summary of measurements from 3 individual assays (mean ± standard deviation). Statistics: two tailed students’ t test. (c) Taking the median value of lncRNA DCST1-AS1 in CRC tissue as the cutoff, 60 patients with CRC were classified as high or low expression group (n = 30 in each group). The overall survival rate in two groups was assessed by Kaplan-Meier survival curve. *P < 0.05, **P < 0.01, and ***P < 0.001

RETRACTED

### Silencing lncRNA DCST1-AS1 inhibits the proliferation, migration, and invasion of CRC cells

To functionally confirm the role of lncRNA DCST1-AS1 in the progression of CRC, lentiviruses carrying shRNA targeting lncRNA DCST1-AS1 (sh-lncRNA DCST1-AS1#1, sh-lncRNA DCST1-AS1#2) were used to stably knock down lncRNA DCST1-AS1, and pcDNA3.1-DCST1-AS1 expression plasmids were used to overexpress DCST1-AS1. HT-29 cell line with high expression of lncRNA DCST1-AS1 was infected with lentiviruses to generate stable lncRNA DCST1-AS1 knockdown, and HCT116 cell line with low expression of lncRNA DCST1-AS1 was transfected with pcDNA3.1-DCST1-AS1 plasmid to overexpress lncRNA DCST1-AS1. According to RT-qPCR results, lncRNA DCST1-AS1 expression level was significantly reduced in both sh-lncRNA DCST1-AS1 #1 and sh-lncRNA DCST1-AS1#2 groups in HT-29 cells, and lncRNA DCST1-AS1 level was dramatically increased after plasmid transfection in HCT116 cells (Figure 2a). CCK8 assay demonstrated that silencing lncRNA DCST1-AS1 in HT-29 cells with both shRNAs restricted the proliferation of cells, while overexpressing lncRNA DCST1-AS1 in HCT116 cells enhanced the cell proliferation (Figure 2b). In addition, colony formation assay and transwell migration assay revealed that knocking down lncRNA DCST1-AS1 inhibited cell colony formation, cell migration, and invasion ability of HT-29 cells. In contrast, lncRNA DCST1-AS1 overexpression promoted the colony formation, migration and invasion of HCT116 cells (Figure 2c-e). In order to further evaluate the role of lncRNA DCST1-AS1 on *in vivo* tumorigenesis, we employed a xenograft tumorigenesis model by subcutaneously injecting HT-29 cells into nude mice. We found lncRNA DCST1-AS1 knockdown significantly suppressed tumor growth (figure 2f). Furthermore, Immunohistochemistry staining demonstrated that silencing lncRNA DCST1-AS1 decreased the level of proliferation marker Ki67 and the mesenchymal marker N-cadherin, but increased the expression of epithelial marker E-cadherin (Figure 2g). Together, these results indicate a functional role of lncRNA DCST1-AS1 in supporting CRC tumorigenesis *in vivo* and *in vitro*.

RETRACTED

**Figure 2.** **lncRNA DCST1-AS1 silencing inhibits cell growth, invasion and migration.** (a) RT-qPCR was conducted to detect lncRNA DCST1-AS1 knockdown efficiency. (b) Proliferation ability of HT-29 and HCT116 cells with lncRNA DCST1-AS1 knockdown or overexpression was assessed by CCK8. (c) The long-term proliferative capacity of HT-29 cells with lncRNA DCST1-AS1 knockdown and HCT116 cells with lncRNA DCST1-AS1 overexpression was analyzed by colony formation experiment. (d) and (e) The migration (d) as well as invasion (e) ability of HT-29 cells with lncRNA DCST1-AS1 knockdown and HCT116 cells with lncRNA DCST1-AS1 overexpression and their control cells were evaluated by transwell experiment. (f) In vivo tumorigenesis analysis of HT-29 cells with lncRNA DCST1-AS1 knockdown or control cells. (g) E-cadherin, N-cadherin and Ki67 expression levels in xenograft tumor tissues were assessed by immunohistochemistry. The above data in A-E are the summary of the measurements of 3 independent experiments (mean ± standard deviation). Comparisons between each treatment and the control were analyzed by the two-sided students’ t-test in a, c, d and e. Repeated-measurement ANOVA was used to analyze B and F. *P < 0.05, **P < 0.01, and ***P < 0.001

### LncRNA DCST1-AS1 acts as a sponge of miR-582-5p in CRC cells

To further explore the mechanism how lncRNA DCST1-AS1 regulates CRC progression, we employed online bioinformatic tool DIANA (http://carolina.imis.athena-innovation.gr/diana_tools/web/) to predict potential miRNA targets of lncRNA DCST1-AS1. We found that hsa-miR-582-5p is ranked as a top miRNA target of lncRNA DCST1-AS1 (Figure 3a **and Figure S1**). In addition, hsa-miR-582-5p has been recognized as a tumor suppressor in prostate cancer (PCa) and non-small cell lung cancer (NSCLC) [23,24]. We therefore selected hsa-miR-582-5p to further investigate its potential interaction with lncRNA DCST1-AS1. DNA fragment containing hsa-miR-582-5p binding site on lncRNA DCST1-AS1 or the fragment with mutated binding site were inserted to pmirGLO (luciferase reporter plasmid) for dual-luciferase reporter assay. HT-29 and HCT116 cells were co-transfected with WT-DCST1-AS1/MUT-DCST1-AS1 luciferase reporter and miR-582-5p mimics/miR-NC. As shown by our assay, hsa-miR-582-5p mimic reduced the luciferase activity of WT-DCST1-AS1 reporter, but had no effect on MUT-DCST1-AS1 group (Figure 3b), which implies that hsa-miR-582-5p can interact with lncRNA DCST1-AS1. We further performed RNA pull-down assay using biotin-conjugated lncRNA DCST1-AS1 probe. LncRNA DCST1-AS1 probe could specifically enrich hsa-miR-582-5p when compared to the control probe, which suggests the physical interaction between miR-582-5p and lncRNA DCST1-AS1 in HT-29 and HCT116 cells (Figure 3c). RT-qPCR analysis further revealed that silencing lncRNA DCST1-AS1 in HT-29 cells significantly upregulated hsa-miR-582-5p, while lncRNA DCST1-AS1 overexpression suppressed hsa-miR-582-5p expression in HCT116 cells (Figure 3d). Consistently, the expression level of hsa-miR-582-5p was significantly lower in clinical CRC tumor tissues than that of normal tissues (Figure 3e). Pearson correlation analysis further revealed a negative correlation between hsa-miR-582-5p and lncRNA DCST1-AS1 expression in CRC tumor samples (figure 3f). Together, the above results suggest that miR-582-5p is a downstream target of lncRNA DCST1-AS1. LncRNA DCST1-AS1 can potentially bind to hsa-miR-582-5p and inhibits its expression.

RETRACTED

**Figure 3.** **lncRNA DCST1-AS1 inhibits hsa-miR-582-5p level within CRC.** (a) hsa-miR-582-5p binding site in lncRNA DCST1-AS1 was revealed using DINAN approaches. (b) Functional interaction between hsa-miR-582-5p and lncRNA DCST1-AS1 was analyzed through the dual-luciferase reporter assay. (c) Physical interaction between hsa-miR-582-5p and lncRNA DCST1-AS1 within HT-29 and HCT116 cells was detected by RNA pull-down assay. (d) hsa-miR-582-5p expression within HT-29 cells with lncRNA DCST1-AS1 knockdown and HCT116 cells with lncRNA DCST1-AS1 overexpression and their control cells were quantified through RT-qPCR. (e) hsa-miR-582-5p levels within 60 CRC samples and matched non-carcinoma samples were analyzed through RT-qPCR. (f) Relationship of hsa-miR-582-5p expression with lncRNA DCST1-AS1 within CRC samples was detected through the Pearson correlation analysis. These data in b-e are the summary of the measurements of 3 independent experiments (mean ± standard deviation). Comparisons between each treatment and the control were measured through two-sided students’ t-test. *P < 0.05, **P < 0.01, ***P < 0.001

We also evaluated the functional role of hsa-miR-582-5p in regulating CRC phenotype. Our data showed that transfection of hsa-miR-582-5p mimic suppressed proliferation (Figure 4a), colony formation (Figure 4b), cell migration (Figure 4c) and cell invasion (Figure 4d) in both HT-29 and HCT116 cells. In contrast, the presence of hsa-miR-582-5p inhibitor promoted proliferation (Figure 4a), colony formation (Figure 4b), cell migration (Figure 4c) and cell invasion (Figure 4d). Together, these findings suggest modulating hsa-miR-582-5p activity regulates CRC cells aggressiveness.

RETRACTED

**Figure 4.** **Hsa-miR-582-5p suppresses proliferation, migration and invasion of cells.** (a) Proliferation ability was assessed by CCK8 assay after cells were transfected with miR-582-5p mimic or miR-582-5p inhibitor or their controls. (b) The colony formation ability was detected by colony formation assay after cells were treated above. (c) and (d) The migration (c) and invasion (d) abilities were evaluated by Transwell assay after cells were treated above. The above data are the summary of the measurements of 3 independent experiments (mean ± standard deviation). Comparisons between each treatment and the control in B-D were measured through two-sided students’ t-test. Comparison between two groups was measured by repeated-measurement ANOVA in A. *P < 0.05, **P < 0.01, and ***P < 0.001

### Hsa-miR-582-5p targets HMGB1 3ʹUTR and regulates its expression in CRC cells

We next sought to identify potential protein target of hsa-miR-582-5p by using TargetScan database (http://www.targetscan.org/vert_72/). We found that there is a binding site of hsa-miR-582-5p on HMGB1 3ʹUTR (Figure 5a), and this binding site seems to be highly conserved among different species (**Figure S2**). Since the HMGB1 act as an oncogenic protein with high expression in different type of cancers [29–33], we further investigated whether hsa-miR-582-5p could regulate HMGB1 expression to mediate the downstream effect of LncRNA DCST1-AS1. We cloned the fragment of HMGB1 3ʹUTR containing the binding site of hsa-miR-582-5p and the fragment with mutated binding site into luciferase reporter vector, and performed dual-luciferase assay by transfecting HT-29 and HCT116 cells with WT-HMCB1/MUT-HMCB1 luciferase reporter and hsa-miR-582-5p mimic/miR-NC. hsa-miR-582-5p could significantly decrease the luciferase activity of WT-HMGB1 group, but showed no effect on MUT-HMGB1 reporter (Figure 5b). RT-qPCR and western blot further demonstrated that hsa-miR-582-5p mimic significantly reduced the mRNA and protein levels of HMGB1 (Figure 5c & Figure 5d). We further analyzed the expression of HMGB1 in paired CRC tumor tissues and the normal tissues. HMGB1 expression level was significantly higher in CRC tumor tissues (Figure 5e). Pearson correlation analysis further revealed a significant positive correlation between the expression levels of HMGB1 and lncRNA DCST1-AS1, while a negative correlation was observed between the expression levels of HMGB1 and hsa-miR-582-5p (figure 5f). Overall, the above results demonstrated that hsa-miR-582-5p can interact with HMGB1 mRNA and negatively regulate its expression.

**Figure 5.** **Hsa-miR-582-5p regulates HMGB1 expression within CRC via targeting HMGB1 3ʹUTR.** (a) hsa-miR-582-5p binding site in HMGB1 3ʹUTR was analyzed using TargetScan database. (b) Dual-luciferase reporter assay was conducted to assess the functional interaction of hsa-miR-582-5p with HMGB1. (c) RT-qPCR was conducted to quantify HMGB1 mRNA level within HT-29 and HCT116 cells after hsa-miR-582-5p over-expression by transfection. (d) WB assay was conducted to assess HMGB1 protein expression within HT-29 and HCT116 cells after transfecting hsa-miR-582-5p. (e) HMGB1 levels within paired CRC samples and non-carcinoma samples were quantified through RT-qPCR. (f) Correlation of hsa-miR-582-5p level with HMGB1 level within CRC tissues was examined through Pearson correlation analysis. The above data in B-D are the summary of the measurements of 3 independent experiments (mean ± standard deviation). Comparisons between each treatment and the control in B-E were measured through two-sided students’ t-test. The correlation between the expression of the two molecules was analyzed by Pearson correlation coefficient analysis in F. *P < 0.05, **P < 0.01, and ***P < 0.001

RETRACTED

### LncRNA DCST1-AS1 regulates the proliferation, migration, and invasion of CRC via miR-582-5p/HMGB1 axis

In order to validate whether hsa-miR-582-5p/HMGB1 axis was involved in lncRNA DCST1-AS1 mediated CRC cell proliferation and motility, we further compared the HMGB1 expression level, cell proliferation, invasion, and migration of different treatment groups (In HT-29 cells: sh-NC, sh-lncRNA DCST1-AS1#1, sh-lncRNA DCST1-AS1#1+ hsa-miR-582-5p inhibitor, sh-lncRNA DCST1-AS1#1+ OE-HMGB1; In HCT116 cells: empty vector, DCST1-AS1 overexpression plasmid, DCST1-AS1+ hsa-miR-582-5p mimic, DCST1-AS1+ HMGB1 siRNA). The results showed that lncRNA DCST1-AS1 knockdown significantly downregulated the expression of HMGB1 and suppressed cell proliferation, migration, and invasion ability when compared to sh-NC group in HT29 cells. The presence of hsa-miR-582-5p inhibitor or HMGB1 overexpression restored the level of HMGB1 (Figure 6a & b), and abolished the inhibition of sh-lncRNA DCST1-AS1 on cell proliferation, migration, and invasion ability (Figure 6c-f). However, in HCT116 cells the overexpression of DCST1-AS1 promoted the HMGB1 expression and aggressive phenotype, which could be attenuated by hsa-miR-582-5p mimic and HMGB1 silencing (Figure 6a-f). Taken together, these results indicate that lncRNA DCST1-AS1 regulates CRC cell growth and motility by modulating hsa-miR-582-5p/HMGB1 axis.

**Figure 6.** **LncRNA DCST1-AS1 regulates CRC cell growth, migration and invasion through the hsa-miR-582-5p/ HMGB1 axis**. HT-29 cells were treated as follows: sh-NC, sh-lncRNA DCST1-AS1#1, sh-lncRNA DCST1-AS1#1+ hsa-miR-582-5p inh, sh-lncRNA DCST1-AS1#1+ OE-HMGB1. HCT116 cells were treated as follows: vector, lncRNA DCST1-AS1, lncRNA DCST1-AS1+ hsa-miR-582-5p mimic, lncRNA DCST1-AS1+ siHMGB1. (a) The HMGB1 mRNA expression were quantified by RT-qPCR. (b) HMGB1 protein levels within HT-29 and HCT116 cells in above experimental groups were detected by western blot. (c) The proliferation ability of HT-29 and HCT116 cells in above experimental groups was assessed by CCK8. (d) Long-term proliferation ability of HT-29 and HCT116 cells in above experimental groups was examined by the colony formation assays. (e-f) Transwell assays (without Matrigel for migration assay; with Matrigel for invasion assay) were performed to assess HT-29 and HCT116 cell migration (e) and invasion (f). The above data in A-F are the summary of the measurements of 3 independent experiments (mean ± standard deviation). Comparisons between two groups were measured through one-way ANOVA in A, B, D, E and F. Repeated-measurement ANOVA was used to analyze C. *P < 0.05, **P < 0.01, and ***P < 0.001

RETRACTED

## Discussion

In this study, we found that lncRNA DCST1-AS1 was significantly upregulated in CRC tissues and cell lines, which was associated with a poorer overall survival of CRC patients. Loss-of-function and gain-of-function experiment in CRC cell lines demonstrated the oncogenic role of lncRNA DCST1-AS1 in promoting the malignant phenotype of CRC cells. We further identified hsa-miR-582-5p as a binding partner of lncRNA DCST1-AS1. By negatively regulating the expression of hsa-miR-582-5p, lncRNA DCST1-AS1 enhances the expression of HMGB1 to promote the aggressiveness of CRC cells. Collectively, our data suggest that lncRNA DCST1-AS1/hsa-miR-582-5p/HMGB1 axis plays an important role in modulating the malignant phenotype of CRC cells.

Emerging studies show that lncRNAs play crucial roles in cell physiology and pathology. LncRNA DCST1-AS1 is suggested to play an oncogenic role in cancer initiation and development. For example, lncRNA DCST1-AS1 promotes the development of cervical cancer (CC) [41], cervical squamous cell carcinoma [42], endometrial carcinoma [43], gastric cancer [44], Triple-negative breast cancer [18] and hepatocellular carcinoma [17] by targeting miRNAs. In our study, we found that the lncRNA DCST1-AS1 is upregulated in CRC tumor tissues, and patients with high level of lncRNA DCST1-AS1 is associated with a poor prognosis. We also detected higher level of lncRNA DCST1-AS1 expression in CRC cell lines when compared to normal human colonic epithelial cells. Those data support the notion that lncRNA DCST1-AS1 acts as a cancer promoting factor in CRC. Our data further demonstrated the requirement of lncRNA DCST1-AS1 in the proliferation, migration, and invasion of CRC cells, which confirms a functional role of lncRNA DCST1-AS1 in promoting the progression of CRC.

RETRACTED

Non-coding miRNA hsa-miR-582-5p has been reported as a tumor suppressor in many malignant tumors to suppress the initiation and development of tumors. Has-miR-582-5p negatively regulates growth and migration of CRC cells [45,46]. Hsa-miR-582-5p has been shown to inhibit the bladder cancer progression [23,47] and its expression is down-regulated in non-small cell lung cancer (NSCLC) tissue [24]. In addition, miR-582-5p is also found to decrease within gastric cancer and it functions to inhibit the proliferation and promote apoptosis of gastric cancer cells [48]. LncRNAs (such as snhg16, pcbp1-as1 and UCA1) can interact with miRNAs (such as miR-198, miR-582-5p) to jointly regulate the development of CRC [49]. However, it remains unclear whether has-miR-582-5p is also regulated by lncRNA DCST1-AS1 in CRC. Our study provided evidence that the expression of lncRNA DCST1-AS1 is negatively correlated with has-miR-582-5p, and they can physically interact with each other. The upregulation of lncRNA DCST1-AS1 could inhibit the expression of has-miR-582-5p, which may account for its oncogenic activity.

HMGB1 has been implicated with tumorigenesis in many studies. In CRC, HMGB1 acts as a tumor-promoting factor to augment the proliferation and metastasis of cancer cells. HMGB1 expression seems to correlate with metastasis of cancer cells and the prognosis of patients [50–52], thus it is suggested that HMGB1 is a possible diagnostic and therapeutic target for CRC [31,32]. HMGB1 expression could be regulated by miRNAs. For example, HMGB1 mRNA level is reported to be negatively affected by miR-129-5p [53]. Our study further revealed that hsa-miR-582-5p targeted HMGB1 3ʹUTR and diminishes the expression of HMGB1. Therefore, HMGB1 is involved in the regulation of CRC progression as a downstream target of hsa-miR-582-5p downstream. Importantly, rescue experiments demonstrated that hsa-miR-582-5p/HMGB1 axis are downstream targets of lncRNA DCST1-AS1 to mediate its oncogenic effects. However, the mechanisms by which HMGB1 regulates the phenotype of CRC cells remains to be further investigated.

In our study, we focused on hsa-miR-582-5p/HMGB1 axis because hsa-miR-582-5p has been previously implicated in the regulation of CRC metastasis [45,46]. On the other hand, HMGB1 was previously reported to promote the proliferation and metastasis of CRC cells [50–52]. However, the regulatory roles of lncRNA DCST1-AS1/miR-582-5p/HMGB1 module has not been previously reported in CRC. This study enriches the regulatory network of lncRNA DCST1-AS1 in CRC and deepens our understanding of the development of CRC. Targeting lncRNA DCST1-AS1 combined with hsa-miR-582-5p/HMGB1 axis may lay a theoretical foundation for targeted therapy for CRC.

RETRACTED

## Conclusion

This study explored and revealed the novel role and mechanism by which lncRNA DCST1-AS1 regulates the aggressive phenotype of CRC cells. The oncogenic factor lncRNA DCST1-AS1 promotes the aggressive phenotype of CRC cells by sustaining CRC cell growth, invasion, and migration. Our results further demonstrated that hsa-miR-582-5p/HMGB1 axis is a downstream target of lncRNA DCST1-AS1. LncRNA DCST1-AS1 interacts and negatively regulates hsa-miR-582-5p, which subsequently maintain the HMGB1 level to support the progression of CRC. Targeting hsa-miR-582-5p/HMGB1 axis can be developed into future therapeutic strategy in controlling CRC progression.

## Supplementary Material

Supplemental Material

## Data statement

Data will be provided on reasonable request.
